This article has been retracted.

# Healthcare and Fitness Data Management Using the IoT-Based Blockchain Platform

**DOI:** 10.1155/2021/9978863

**Published:** 2021-07-09

**Authors:** Tarek Frikha, Ahmed Chaari, Faten Chaabane, Omar Cheikhrouhou, Atef Zaguia

**Affiliations:** ^1^Université de Sfax, CES Lab, Sfax, Tunisia; ^2^Université de Sfax, REGIM Lab, Sfax, Tunisia; ^3^College of Computers and Information Technology, Taif University, Taif 21944, Saudi Arabia

## Abstract

Because of the availability of more than an actor and a wireless component among e-health applications, providing more security and safety is expected. Moreover, ensuring data confidentiality within different services becomes a key requirement. In this paper, we propose to collect data from health and fitness smart devices deployed in connection with the proposed IoT blockchain platform. The use of these devices helps us in extracting an amount of highly valuable heath data that are filtered, analyzed, and stored in electronic health records (EHRs). Different actors of the platform, coaches, patients, and doctors, collaborate to provide an on-time diagnosis and treatment for various diseases in an easy and cost-effective way. Our main purpose is to provide a distributed, secure, and authorized access to these sensitive data using the Ethereum blockchain technology. We have designed an integrated low-powered IoT blockchain platform for a healthcare application to store and review EHRs. This architecture, based on the blockchain Ethereum, includes a web and mobile application allowing the patient as well as the medical and paramedical staff to have a secure access to health information. The Ethereum node is implemented on an embedded platform, which should provide an efficient, flexible, and secure system despite the limited resources and low power consumption of the multiprocessor platform.

## 1. Introduction

Despite all the efforts made and the shields raised to achieve the security purpose, technological evolution has not ceased to create loopholes that have always been used to attack, hack, and control these systems.

Among the new technologies aimed at information security, the blockchain cannot be overlooked. Indeed, the use of this technology has made it possible to minimize dependence on a third party while increasing the security of users. One of the main fields guessing more and more security is the e-health one, which needs to highly preserve the medical data.

In this context, our paper presents a hybrid e-health approach that allows the implementation of a decentralized system. This system helps to enhance security and privacy of medical, paramedical, and personal data with less confidentiality.

Aiming at a low-consumption system, we call upon the blockchain Ethereum to realize an e-health platform.

The contribution of this paper is as follows:

- Implementation of a secure, hybrid, medical, and paramedical application based on the Ethereum blockchain
- Improvement in the architecture of the blockchain nodes to reduce power consumption
- Implementation of a web and mobile platform to access and add data to the blockchain

The remainder of this paper is as follows. First, we will start with a blockchain overview and then the state of the art on the blockchain applications and e-health blockchain application in particular. In Section 4, we propose a secure e-health application through the use of the blockchain. In Section 5, we propose a general description of application implementation. It contains different Ethereum blockchain implementations' part and the used mobile and web application. Finally, we conclude the paper with a conclusion and some perspectives.

## 2. Blockchain Overview

Blockchain is an information storage and distribution technology that is transparent and secure and operates regardless of a central control body.

Let us take the example of two users of blockchain ∝_1 and ∝_2, 2 out of *N* users in an end-to-end network in which the exchange of messages is based on an authenticated and decentralized way. The messages sent by ∝_1 to ∝_2 are first authenticated by one or a group of users in the network, according to a consensus protocol. Once authenticated, the message is stored (based on the IDs of ∝_1, ∝_2, and the authenticator) in an archive that is distributed to all network users. Assuming that a malicious user or group of users wants to modify the local copy of the archive, other users can easily identify the malicious user or group of users and correct the modification accordingly.

The blockchain can, therefore, be likened to a database that contains the history of all exchanges between different users since it was set up. This database is secure and distributed: it is shared by its different users, without intermediaries, which allows everyone to check the validity of the chain [1].

Transactions between network users are grouped into blocks. Each block is validated by the network nodes. These nodes are called “minors.” Once validated, the block is added to the blockchain. The transaction is then visible to the receiver as well as to all users of this network.

Blockchain is based on asymmetric cryptography, also known as public key infrastructure (PKI) [2], which uses a key pair (a public key and a private key) to encrypt and decrypt the data. The keys are paired hands which are not identical (asymmetric).

We can summarize the advantages of the blockchain in 5 parts which are as follows [3]:

- Trustless: as mentioned earlier, the decentralization of information means that the exchange of information takes place without the need for a trusted third party.
- Reliability: the importance of decentralization as stated in trustless eliminates the problem of the central point. This minimizes the risk of succumbing to attacks.
- Integrity: transaction execution is done like a command protocol. This allows it to have integrity.
- Transparency: the transparency of the blockchain is apparent in the fact that any changes made to the public channels are public and can be analyzed and accessed by all members of the blockchain, hence the transparency.
- Quality data: the blockchain's data are complete, consistent, and unchangeable.

In this section, we have presented the blockchain and its features and benefits. In the following part, we will describe different blockchain components.

(i) Transactions: these are the exchanges of data between different users. Each transaction is signed by the sender's private key. Thanks to this signature, the security of the transactions is guaranteed. Therefore, any modification of these transactions during transmission can be avoided.
(ii) Blocks: a block is a record in the blockchain which contains the confirmed transactions. Thus, each open transaction will be added to a block. After a period of time, in order for a new block containing transactions to be added to the blockchain, it must be validated by a selected person called a minor. This validation operation is called minage.
(iii) Blockchains: each block in the blockchain is linked to the previous block. This link is done by inserting the hash specific to the previous block. Therefore, the hash of each block includes not only its own hash but also the hash of the previous block.  Figure 1 illustrates what has been described. This way, we can protect our blockchain from any form of corruption. This prevents any modification of the content of the existing blocks.
(iv) Smart contracts: a smart contract is software “installed” on a blockchain solution. It is the most important link in our blockchain. It runs automatically as soon as various preprogrammed constraints are checked. Despite the fact that it is not a legal document per se, the intelligent contract automates the execution of a contractual commitment.
(v) In order to choose which blockchain framework to use, it is important to define characteristics that allow comparison between different frameworks. Among the blockchain criteria are consensus mechanisms, smart contracts, permissioned blockchains, layer of services, M2M blockchain applications, and mobile compatibility [5].
  - The consensus mechanism (C.M):
  - A consensus algorithm is a process through which all the nodes of the blockchain network achieve a common agreement about the actual state of the distributed ledger [6]. A well-designed consensus protocol can ensure the fault tolerance, authenticity, and security of a blockchain system. Several protocols exist today, but the most used are proof of work (PoW), proof of stake (Pos), and proof of authority (PoA) which is a more recently created protocol than both PoW and PoS.
  - Proof of work:
  - The proof of work (PoW) consensus mechanism is the most adopted consensus mechanism in existing blockchains. PoW was first used by bitcoin and presumes every peer vote with his “hashing power” by solving proof of work puzzles and creating the appropriate blocks [7, 8].
  - Proof of authority:
  - Proof of authority (PoA) is a family of consensus protocols for permissioned blockchains whose notoriety is due to performance boosts with respect to conventional BFT algorithms. PoA protocols count on a set of *N* trusted peers known as the authorities. Each authority is recognized by a unique ID, and most of them are believed to be honest, that is, at least *N*/2 + 1. The authorities achieve a consensus to validate and sign the transactions issued by clients [9].
  - Smart contracts (S.C):
  - As described earlier, some blockchains use smart contracts, others do not support them, while the latter type of blockchain uses decentralized applications.
  - Permissioned blockchains (P):
  - This is the ability to designate different roles and rights to be given to the nodes of the blockchain.
  - Layer to services (L2S):
  - A layer to service should be able to retain decentralized benefits while scaling the transaction capacity of the digital ledger. It permits to choose between supporting 1 service and 2 services.
  - M2M blockchain applications (M2M B.A):
  - allows one to check the blockchain's suitability for machine-to-machine (M2M) applications. This makes it easier to use different applications of the IoT [10].
  - Mobile compatibility (M.C):
  - Using mobile systems with limited resources has become increasingly common. As a result, it allows smartphones not only to belong to the blockchain network but also to run a node. It is also possible to run the same type of work as a traditional node [11].

As part of this work, we chose to implement a health application based on the medical and physical data of the users. These data will be stored using a secure application based on the blockchain.

With the evolution of the blockchain, several platforms have emerged. We can cite Ethereum [12], Tezos [13], IOTA [14], Hyperledger Fabric [15], and Enigma [16].

In Table 1, we compare different blockchains using consensus mechanisms (C.M), smart contracts (S.C), permissioned blockchains (P), layer to services (L2S), M2M blockchain applications (M2M B.A), and mobile compatibility (MC) as features.

Although IOTA appears to be the most malleable blockchain, Ethereum provides the flexibility to choose between different consensus protocols and therefore run the network on a light multiprocessor architecture, and the one most used in the industry remains Ethereum. This is why we chose to use Ethereum [3].

In this paper, we will adopt the blockchain Ethereum with the M2M layer. The application that will allow us to highlight this will be the e-health application that will be presented in Section 3.

The use of the blockchain, which was exclusive to the financial sector, has become widespread [17]. Some of the areas of the use of the blockchain are the following:

  Stock market [18]
  Energy industry [19]
  Insurance [20]
  Healthcare [4, 21, 22]
  P2P multimedia content distribution platforms [23, 24]

In this section, we have presented a description of the blockchain. Treating an application related to the health field, we will make a state of the art on the work of blockchain applied to e-health.

## 3. State of the Art: Blockchain for the E-Health Application

The healthcare industry confronts the third evolutionary trend of IT digital technologies with implications, so profound analysts think it is a new era of global computing [25]. Indeed, for all organizations, digital transformation will be galvanized by foundational technologies such as mobility, 3D [26], Internet of Things (IoT) [27], big data, deep learning [28, 29], machine learning [30] using segmentation [31] and classification process [32–34], and Healthcare 4.0 [35, 36] coming from Industry 4.0 [37, 38].

Health technologies [39] have improved continuously ever since the early stages of medicine. Ever-increasing knowledge, diagnostic, preventive treatment, and rehabilitation opportunities have altered the matter of healthcare systems. The “digital transformation of health services” is seen as a crucial and influential process that has already had substantial bearing on current healthcare and health systems and is believed to have a further fundamental influence on healthcare and healthcare delivery in the future.

Many research studies and projects have dealt with the use of the blockchain technology and IoT in e-health systems. More and more healthcare organizations are applying the blockchain technology in their systems; this technology is playing a crucial role in the healthcare market nowadays [40]. It can provide automated data gathering and verification processes, accurate and accumulated records from different sources which are immutable, tamper proof, and offer safeguarded data, with a lower risk of cyberattacks. Currently, the healthcare business faces different challenges regarding the security incidents, data integrity, data ownership, etc.

Electronic health record systems make healthcare services more efficient. They can reduce the significant workload of the clinician and provide diagnostic assistance that helps prevent medical errors [41]. They can document diagnostic investigations and medical treatments, provide clinical decision support, and facilitate communication among healthcare providers [42].

In [40], Tanwar et al. presented a system based on Healthcare 4.0 application. The blockchain technology offers a system architecture that guarantees secure access to data with an access control policy implemented for participants to achieve privacy and data ownership for patients in the EHR system.

Dagher et al. [43] proposed a privacy-preserving framework for access control and interoperability of electronic health records using the blockchain technology. The proposed framework, implemented over the existing system, is based on Ethereum. It uses encryption and authentication throughout the blockchain, which demonstrates the prioritization of security and access control.

The proposed architecture removes the central authority and does not present a single point of failure in the system, thanks to the distributed nature of the blockchain. System security is reached, thanks to the immutability of the decentralized ledger as any node cannot alter the ledger. Using a less power consumption consensus network that can validate transactions and mint blocks in a fast and secure way shows the blockchain's potential and significance in several areas and confirms that it could be the next revolutionary technology for proposing new healthcare system architectures.

Several works have presented different directions of research orientation in the field of blockchain applied to healthcare. In [44], Khezr et al. proposed various blockchain applications in the healthcare industry and identified the major research initiatives as well as future research opportunities. They presented current research on health data management and how blockchain will empower patients and streamline the sharing process of the health data. A description of a consensus among researchers is that, with blockchain technology, patient data will be truly owned and controlled by the patient himself. The blockchain allows for health records to be time-stamped so that no one can tamper with them after becoming part of the distributor ledger. This is why the patients will have the right to decide who can and cannot access to their data and for what purpose. The proposed approach is based on confidential health data.

In order to permit patients to gain control over their health data by reducing the fragmentation of information, a patient-centric health data-sharing framework called MedChain was proposed by Shen et al. [45]. This work showed that it was more efficient for sharing data without compromising security, thanks to a dual-network architecture, a session-based data-sharing system, and a condensed chain structure. At the same time, the scope of the healthcare data is being expanded to include data streams from various monitoring devices, which can further assist physicians and medical researchers. Hence, MedChain can maximize the interest of all parties, and the result is significant as efficiency has been proven to be one of the main issues in the adoption of the healthcare chain.

While most of the works propose approaches to secure critical medical information that can only be accessed by physicians, patients, or, in some cases, healthcare providers or retailers, our application presented in this paper is a hybrid e-health application that includes data that must remain confidential and accessible to physicians, while other data can be shared by other actors.

The need for a shared distributed environment based on trust shows the value of using the blockchain to provide this trust. The proposed approach for our low-power hybrid application is presented in Section 4.

## 4. The Proposed Approach for a Healthcare Application

In our model, we focus on a patient-centric application for storing electronic medical records. For this purpose, we assume that the patient is using some wearable devices capable of continuously measuring a predefined set of parameters of the health status of the patient (such as calories, oxygen saturation, heart rate, and hypertension). The data gathered by these wearable sensors are permanently uploaded to the decentralized ledger. These data are also stored to retrieve back the patient's status development, allowing the healthcare personnel to have better visibility of his evolution. All the interactions between different actors of our use case handle very sensitive personal data. Therefore, it is crucial that these medical records must remain confidential and have limited and controlled access in our system which guarantees the nonrepudiation of the records. Our architecture's design aims to satisfy all these requirements through the use of the blockchain technology to hold electronic health records.

Figure 2 shows our architecture. It is mainly composed of wearable devices that synchronize the data with a mobile application and a web application, allowing healthcare personnel to monitor their patients.

### 4.1. Wearable Device

Each patient should be equipped with one or more wearable devices capturing a set of health parameters that define the patient's status (such as heart rate, calories, distance, steps, and temperature). This device synchronizes the data with the mobile application through Bluetooth.

### 4.2. Mobile Application

This application is installed on the patient's mobile phone; it enables him to create a wallet (containing his public and private key) and to deploy his own smart contract to the Ethereum network. The application reads the health data from the wearable device and stores them in the patient's smart contract. The data upload to the blockchain could be on demand or a task that runs every day, every 2 hours, depending on the patient's configuration.

### 4.3. Smart Contract

In our architecture, each patient is supervised by a wearable device. This device is in charge of gathering data that will be stored in the patient's smart contract. Hence, for each patient, one smart contract is deployed. The use of the smart contract is explained in the following section.

### 4.4. Web Application

It is the entity that visualizes data continuously and allows health professionals to monitor the patient's status depending on their access level.

### 4.5. Health Professional

He can be a doctor, a nutritionist, a physicist, etc. He represents a node in our blockchain network. He can visualize the data through the web application based on the stored data. These data are stored in a database in the cloud. At each registration, the transaction must be confirmed and subsequently saved in the smart contract.

Health professionals are divided into two groups:

- The patient's doctors who have the ability to view and add information about the patient via the blockchain. They have access to various medical information.
- The health actors such as the physiotherapist, the sports coach, and the nutritionist to whom some data are accessible while others are confidential. These actors have the right to add information via their blockchain node.

### 4.6. Patient

He is not a node in the blockchain network; he only interacts with it through his mobile phone, receiving data from the wearable devices and sending them to the blockchain to be stored in the smart contract.

In the following sections, the implementation of our architecture will be described in detail.

## 5. Proposed Implementation

In order to implement our architecture, we choose the Ethereum network since it respects the criteria of our requirements. In fact, Ethereum supports the implementation of smart contracts and offers the possibility to choose between different consensus protocols, PoW and PoA.

The PoW offers a secure e-health system that can secure even a public network. One of the major problems of PoW is the need to have significant hardware resources to meet the computational needs.

PoA permits to develop a private and permissioned blockchain with low energy consumption.

### 5.1. Patient's Smart Contract Configuration with Ethereum

Figure 3 shows how we configure the patient's smart contract illustrated in our approach using the Ethereum network.

The proposal request (transaction proposal), which holds to the data obtained from the wearable device, is sent to validating peers (miners) in the network to approve the transaction and add the value to the smart contract. Then, according to the consensus protocol, the validating peers decide whether a transaction is valid or not. If it is valid, the peers sign the transaction and add it to the new block. When the transaction is validated, the new health information entry is stored in the smart contract, and the mobile application is notified of the success of the transaction.

### 5.2. Algorithms

We validate our approach at a design level by running two applications. The first application runs on the patient's mobile phone to sync data with the wearable device and upload them to the blockchain, and the second one is web application that enables health professionals to visualize health information.

#### 5.2.1. Algorithm 1: Upload Data

The algorithm description shown in Figure 4 represents the process of storing the patient data in the blockchain network.

When the user requests to synchronize the data with his wearable device and upload them to the blockchain, first, the mobile application will get the health information from the wearable device and visualize it to the patient. After that, it will execute the smart contract function, as described in Figure 4, which uploads the data which would create a transaction and sends it to the blockchain network in order to be validated by the peers. These latter verify the transaction according to the consensus protocol being used. A response is then given by the peers, whether they validated and signed the transaction or they judged to be unauthentic. With this response, the smart contract and therefore the application will be notified, and the new data entry will be added to the smart contract.

#### 5.2.2. Algorithm 2: Visualize Data

The algorithm description in Figure 5 provides a detailed description of how our application handles visualizing and monitoring the health information of patients by health personnel.

The health professional must connect to the web application in order to monitor his patient's information. Then, he will be redirected to the patients' list where he will find a list of all patients that authorized him to access their data. We used NodeJs and ExpressJs to develop the server side since this approach is more scalable and secure. The web application will request the patient information from his smart contract using the health professional Ethereum credentials. The smart contract will verify that this request is authorized and will give a response that corresponds to the health professional access level, as shown in Figure 5. If the request is authorized, the data will be visualized to the dashboard page.

### 5.3. Running the Ethereum Blockchain

In our model, we chose to work on a private Ethereum blockchain in order to guarantee the safety of the information being stored in smart contracts. To create our own blockchain, we need to define some parameters such as the consensus protocol and number of peers. Furthermore, running these blockchain nodes requires computational power and storage. In this section, we explore and explain the choices we made.

The main idea is to implement an embedded multiprocessor system to support one node of the Etherum blockchain and to meet the low consumption constraint.

Already being implemented on GPU and server-based systems, the blockchain is already fully satisfactory. However, such platforms still consume a lot of energy. Aiming to study the feasibility of implementing Ethereum on multiprocessors which are low-power platforms, an attempt was made to test the feasibility on a platform with 4 ARM processors.

This platform must also offer connectivity, allowing communication with peripherals as shown in Figure 2. Our embedded system must not only be connected to the server but also to the mobile application. Therefore, the presence of Bluetooth and Wifi/3G connectivity is very important.

Among the platforms meeting these constraints, we can mention Raspberry Pi 3. This platform can show us not only the feasibility of the system but also the possible HW improvements that could be made to our architecture as depicted in Figure 2.

#### 5.3.1. Consensus Protocol

When creating an Ethereum blockchain, we can choose between two different consensus algorithms:

- Proof of work
- Proof of authority

In Table 2, we compare different features and characteristics of the proof of work consensus and the proof of authority consensus.

The proof of authority offers faster transactions with lower energy consumption, but it relies on the honesty of its authorities, while the proof of work is a trust-free consensus that is widely deployed and proven to be resilient. In the following section, we will attempt to run two blockchains using both protocols.

#### 5.3.2. Executing the Blockchain

In this section, we will discuss the results of executing a private Ethereum blockchain using each consensus.

- Proof of work:
- After writing our genesis file, running the init command on Raspberry Pi 3 to initialize our blockchain was successful. Then, we were able to execute the node and access the JavaScript console where we performed some basic Ether transfer transactions between the predefined accounts which were successfully submitted, but the moment the miner is being started, RPi3 would overheat and stop functioning. For this, we executed another node from the same blockchain on the computer that was able to mine the transactions and synchronize the results with the node running on RPi3 as illustrated in Figure 6. Therefore, using the proof of work, RPi3 can only synchronize the mined blocks but not mine new ones.
- Proof of authority:
- After writing our genesis file and defining PoA (clique) as our consensus, we defined our sealer accounts as well; running the init command on Raspberry Pi 3 to initialize our blockchain was successful. Then, we were able to execute the node and access the JavaScript console where we performed some basic Ether transfer transactions between the predefined accounts which were successfully submitted. Unlike with PoW, RPi3 was able to mint blocks and validate our transaction using the proof of authority consensus. A second node belonging to this blockchain was executed on the computer as shown in Figure 7.

In this model, RPi3 is the one minting blocks and validating the transaction sent by the client running on the computer. Both nodes will synchronize the actual state of the blockchain. Hence, PoA is more suitable to run on such low computational multiprocessor architecture.

### 5.4. Achievement: Dashboard Interfaces

The key aspect of our project is to visualize data related to a patient while storing them in a secure and confidential way, not only the last entry but also the patient's history since he started using our application. After successful authentication, the patient has the privilege to connect to his wearable device and sync data using his mobile application and eventually upload these data to the smart contract. Furthermore, he may add a health professional (doctor, nutritionit, coach, etc.) in order to give him access to his data.

#### 5.4.1. Mobile Application

The graphical user interface (GUI) as illustrated in Figure 8 contains the following parts:

- Home page: in this, the user will be able to check his health data (heart rate, calories, steps, and distance). The patient has 3 options, sync data with the wearable device without uploading them to the smart contract, sync and upload, or he can also set a recurrent task (for example, it runs every four hours, every day) that syncs the data and send them to the blockchain.
- Account page: it represents the available information related to the patient.
- Add health professional page: in this page, a list of health professionals is shown to the patient. In Figure 9, we can see a list of doctors; the patient can click on the plus button in order to add a doctor to his account and therefore grant him access to his data.

#### 5.4.2. Web Application

The web application consists of two main screens:

  Patients' list: this screen is illustrated in Figure 9. After the health professional is successfully authenticated to the web application, a list of all his patients will be displayed. For a more detailed overview of the patient, the health professional needs to click on the patient he wishes to monitor.
  Patient overview: after clicking on a certain patient, the health professional is directed to the more detailed overview as we can see in Figure 10. In this case, the health professional is connected as a doctor; hence, he has access to all the information, and he is able to check all the charts available.

## 6. Discussions

Compared to the existing works, the proposed platform has improved the security aspect of shared data.

Indeed, regarding the application side, we notice that the blockchain applications touch either the very sensitive and secure medical care or the professional sports section via the less secure physical and nutritional data.

Within the framework of our application, we have succeeded in putting forward a hybrid system that allows both presentation of highly secure confidential medical data and less secure medical data available to certain members who have access to the blockchain. Data related to coaches, physiotherapists, or dieticians are less secure but are only accessible to blockchain members.  Table 3 presents this comparison.

As shown in Table 3, our work presents a heterogeneous multidata, multidisciplinary platform compared to the existing platforms of the state of the art.

The main purpose of the proposed platform is to implement blockchain nodes on a platform with limited resources playing the role of the blockchain support and web server.

From the performance point of view, we try to present the characteristics of the realized system in Figures 6–8. In this part, we will illustrate the obtained results in terms of the number of nodes and energy consumption. Our support platform is Raspberry Pi 3.

Despite its technical limitations tied to limited resources, the use of the Raspberry Pi 3-based platform shows that the proposed approach allows to implement more than one node on Raspberry Pi 3 using PoA as consensus, but it is impossible to mine using PoW when considering its high time and energy consumption.  Table 4 describes different architectures implemented as well as the energy consumption obtained.

It is important to point out that we managed to implement 6 nodes of blockchain Ethereum with PoA. On the consumption side, Raspberry consumes less than 2.3 W for one node and approximately 4.5 W for 6 nodes. The use of PoW as indicated above reaches 5.1 W. If we were using a GPU platform (Jetson TX1), we would need approximately 15 W of power consumption. The best compromise is to choose Raspberry Pi 3 with PoA in order to minimize energy consumption.

## 7. Conclusion

In this paper, we focused on storing electronic health records where the data collected by the deployed devices are critical. Our goal was to offer a distributed, secured, and permissioned access to these sensitive data using the emerging blockchain technology. In this study, we designed an IoT blockchain-embedded architecture for a healthcare application to store and examine EHRs. We explored different blockchain tools and platforms available, and Ethereum was the most adequate to implement our architecture. In order to validate our approach, real applications were executed to demonstrate the functionalities and features of our architecture. As future work, we hope to implement an industrial system. This system should support a wider range of sensors that can be implemented on a wearable device. It offers health personnel more parameters to assess patients. Also, adding a second layer of security by encrypting the data before storing in the blockchain would increase the resilience of our architecture. The second axis proposes to implement our node using the proof of work. Indeed, using codesign allows us to propose a multiprocessor system based on IPs. This system will allow to accelerate the energy-consuming computational part by using several IPs.

## Figures and Tables

**Figure 1:** Illustration of a blockchain [4].

**Figure 2:** EHR storing and monitoring architecture.

**Figure 3:** Patient's smart contract configuration with Ethereum.

**Figure 4:** Upload electronic health records.

**Figure 5:** Read electronic health records.

**Figure 6:** Private Ethereum blockchain using PoW.

**Figure 7:** Private Ethereum blockchain using PoA.

**Figure 8:** Mobile application GUI.

**Figure 9:** Patients' list page.

**Figure 10:** Patient overview page.

**Table 1:** Comparison between the main blockchain platforms.

	C.M	S.C	P	L2S	M2M B.A	MC
Ethereum	No	Yes	No	No	No	No
Tezos	No	Yes	No	No	No	No
IOTA	Yes	Yes	Yes	No	Yes	No
Hyperledger Fabric	Yes	Yes	No	No	No	No
Enigma	No	Yes	No	No	No	No

**Table 2:** Comparison between PoW and PoA properties.

	PoA	PoW
Permissioned blockchains	Yes	No
Private	Yes	No
Energy consumption	Low	High
High processing power needed to create blocks	No	Yes
Risk of 51% attack: network takeover	Low	High
Trust-free	No	Yes
Transaction time	Fast	Slow

**Table 3:** Different fields of blockchain applications.

	Health data	Pharmaceutical data	Sportive data	Physiotherapists' data	Dieticians' data	IoT devices
Shahnaz et al. [4]	Yes	No	No	No	No	No
Dziak et al. [25] and Khezr et al. [44]	Yes	No	No	No	No	Yes
Khezr et al. [44]	Yes	No	No	No	No	Yes
Jamil et al. [46]	Yes	Yes	No	No	No	No
Mulyati et al. [47]	No	No	Yes	No	No	No
Our approach	Yes	No	Yes	Yes	Yes	Yes

**Table 4:** Different architectures and platform implementation.

	Web server	Node number	Energy consumption (W)
RPi3 with PoW	Yes	No nodes	5.1
RPi3 with PoA	Yes	1 node	2.3
		Up to 4 nodes	4.5
Jetson TX1 with PoW	Yes	2 nodes	15
Jetson TX1 with PoA	Yes	More than 10 nodes	15

## Data Availability

No data were used to support this study.
